The article "Propylene Glycol Caprylate-Based Nanoemulsion Formulation of Plumbagin: Development and Characterization of Anticancer Activity" was published in 2022. Journal: Biomed Res Int.

# Propylene Glycol Caprylate-Based Nanoemulsion Formulation of Plumbagin: Development and Characterization of Anticancer Activity

**DOI:** 10.1155/2022/3549061

**Published:** 2022-01-10

**Authors:** Adrian Chrastina, John Welsh, Per Borgström, Veronique T. Baron

**Affiliations:** ^1^Proteogenomics Research Institute for Systems Medicine (PRISM), 505 Coast Blvd. South, La Jolla, CA 92037, USA; ^2^Vaccine Research Institute of San Diego (VRISD), San Diego Science Center, 3030 Bunker Hill, San Diego, CA 92109, USA

## Abstract

Plumbagin, a bioactive naphthoquinone, has demonstrated potent antitumor potential. However, plumbagin is a sparingly water-soluble compound; therefore, clinical translation requires and will be facilitated by the development of a new pharmaceutical formulation. We have generated an oil-in-water nanoemulsion formulation of plumbagin using a low-energy spontaneous emulsification process with propylene glycol caprylate (Capryol 90) as an oil phase and Labrasol/Kolliphor RH40 as surfactant and cosurfactant excipients. Formulation studies using Capryol 90/Labrasol/Kolliphor RH40 components, based on pseudoternary diagram and analysis of particle size distribution and polydispersity determined by dynamic light scattering (DLS), identified an optimized composition of excipients for nanoparticle formulation. The nanoemulsion loaded with plumbagin as an active pharmaceutical ingredient had an average hydrodynamic diameter of 30.9 nm with narrow polydispersity. The nanoemulsion exhibited long-term stability, as well as good retention of particle size in simulated physiological environments. Furthermore, plumbagin-loaded nanoemulsion showed an augmented cytotoxicity against prostate cancer cells PTEN-P2 in comparison to free drug. In conclusion, we generated a formulation of plumbagin with high loading drug capacity, robust stability, and scalable production. Novel Capryol 90-based nanoemulsion formulation of plumbagin demonstrated antiproliferative activity against prostate cancer cells, warranting thus further pharmaceutical development.

## 1. Introduction

Plumbagin (5-hydroxy-2-methyl-1,4-naphthoquinone, Figure 1) is a naturally occurring 1,4-naphthoquinone found in Plumbaginaceae and other plant families [1]. Plumbagin has a variety of pharmacological properties that include potent antitumor, antiatherosclerotic, anti-inflammatory, antibacterial, antifungal, and neuroprotective activities [1–3]. It has demonstrated broad-spectrum anticancer efficacy on diverse types of cancer, including glioma, hepatocellular carcinoma, melanoma, and promyelocytic leukemia, as well as breast, esophageal, lung, ovarian, and prostate cancer [4].

Numerous investigations have indicated that the anticancer activity of plumbagin is mediated through effects via several signal transduction pathways or targets, including AMPK, CDK1/CDC2, cyclin B1, cyclin D1, FOXM1, NF-*κ*B, p53, p21 Waf1/Cip1, p27 Kip1, PI-5, Nrf2/ARE, PI3K/AKT/mTOR, Ras, Sirt1, STAT3/PLK1/AKT, and Wnt [3]. Furthermore, plumbagin is an efficient generator of reactive oxygen species (ROS), inducing oxidative stress in tumor cells [5, 6]. These activities contribute to the anticancer effects of plumbagin, leading to cell cycle arrest and apoptotic death of tumor cells or inhibition of metastatic activity [2].

The article "Propylene Glycol Caprylate-Based Nanoemulsion Formulation of Plumbagin: Development and Characterization of Anticancer Activity" was published in 2022. Journal: Biomed Res Int.

Thus, plumbagin is a promising drug that has drawn a significant interest in anticancer research, leading to the preclinical development of a new therapeutic drug, currently in clinical trial for the treatment of prostate cancer. Initial studies of the effect of plumbagin in prostate cancer came from Dr. Verma's group, which showed that plumbagin inhibited tumor growth rate or significantly delayed disease progression in various models of prostate cancer [7–9]. A key finding from our group showed that plumbagin significantly improved the efficacy of androgen deprivation therapy (ADT) in hormone-responsive models of prostate cancer, leading to tumor regression and extended survival when used in combination with ADT [10, 11]. These preclinical studies established the framework for the first-in-human clinical trial of the combination of plumbagin and ADT in prostate cancer patients (NCT03137758).

Clinical studies of plumbagin, however, have been impeded by its poor solubility in water. Indeed, the rate and extent of a drug absorption and bioavailability following per-oral administration are greatly affected by its solubility [12], and successful clinical deployment of plumbagin will require a formulation that considerably increases its solubility. Therefore, we have developed and characterized a new nanoemulsion-based drug delivery system of plumbagin. Nanoemulsions are biphasic dispersions of oil in water stabilized by amphiphilic surfactant/cosurfactant interfacial film exhibiting optical isotropy and kinetic stability [13]. Particle size of nanoemulsions is typically within the submicron range, 5-200 nm [13]. Importantly, nanoemulsion formulations have critical advantages for oral drug delivery, including high encapsulation capacity and high surface-to-volume ratio, as well as favorable physicochemical properties facilitating their stability. They have been shown to improve drug pharmacological profiles, reducing toxicity, and potentially improving the stability and pharmacokinetics of encapsulated drugs [14, 15].

This study describes the formulation of nanoemulsions using biocompatible components, with propylene glycol caprylate (Capryol 90) as an oil phase and Labrasol/Kolliphor RH40 as surfactant/cosurfactant excipients. High loading capacity for plumbagin, long-term stability, retention of particle size in simulated physiological environments, and increased sensitivity to the antiproliferative activity of plumbagin in prostate cancer cells indicate that Capryol 90-based nanoemulsion formulations of plumbagin are suitable for further development.

The article "Propylene Glycol Caprylate-Based Nanoemulsion Formulation of Plumbagin: Development and Characterization of Anticancer Activity" was published in 2022. Journal: Biomed Res Int.

## 2. Materials and Methods

### 2.1. Materials

Capryol 90 (propylene glycol caprylate), Labrasol (PEG-8 caprylic/capric glycerides), Labrafil M 1944 CS (mono-, di-, and triglycerides and PEG-6 mono- and diesters of oleic acid), Labrafac lipophile WL 1349 (triglycerides of caprylic and capric acids), and Peceol (glyceryl monooleate) were purchased from Gattefosse (Saint-Priest, France). Capmul MCM (mono-diglyceride of caprylic and capric acid) and Capmul PG-12 (propylene glycol monolaurate) were supplied by Abitec Corporation (Columbus, OH). Glyceryl trioleate, Kolliphor RH40 (polyoxyl 40 hydrogenated castor oil), Span 80 (sorbitan monooleate), Span 85 (sorbitan trioleate), plumbagin, and other chemicals were supplied by Sigma (St. Louis, MO).

### 2.2. Determination of Plumbagin Solubility in Pharmaceutical Excipients

The solubility of plumbagin in a series of lipid-based pharmaceutical excipients was determined by UV-VIS spectrophotometry as described previously [16, 17]. Briefly, supersaturated dispersions of plumbagin in excipients were incubated at 25°C for 72 h on a rotary shaker. Samples were centrifuged at 10,000 × g for 10 min, and for each sample, the supernatant was filtered through a syringe filter (0.45 *μ*m). Aliquots of filtrates were dispersed in 200–3000-fold volume excess of methanol. The concentration of plumbagin was determined using absorption spectrophotometry (DU-640 spectrophotometer, Beckman Coulter, Fullerton, CA) with molar absorption coefficient for plumbagin determined in methanol, *ε*_*λ*_ (410 nm) = 3,800 dm^3^·mol^−1^·cm^−1^).

### 2.3. Construction of Pseudoternary Phase Diagram

A pseudoternary phase diagram was generated as described previously [18] by water titration of mixtures of Capryol 90 and increasing amounts of the Labrasol/Kolliphor R-H40 surfactant/cosurfactant blend at 25°C, in concordance with the common requirements for preparation, storage, and application of nanoemulsions. To identify the nanoemulsion domain, the mixtures were visually inspected for clarity to delineate boundaries of phases and further characterized by dynamic light scattering as described below. Particle size distribution was measured directly without further dilution.

The article "Propylene Glycol Caprylate-Based Nanoemulsion Formulation of Plumbagin: Development and Characterization of Anticancer Activity" was published in 2022. Journal: Biomed Res Int.

### 2.4. Particle Size Analysis

Particle size distribution and polydispersity of emulsified formulations were determined by dynamic light scattering (DLS) using noninvasive back scatter (NIBS) detection at a 173° angle and at 25°C on Zetasizer Nano-ZS (Malvern Instruments) equipped with 4 mW He-Ne, 633 nm laser. *Z*-average size (nm) or harmonic intensity averaged particle diameter was calculated by cumulant analysis of autocorrelation function generated from DLS measurement as defined by ISO 13321 and ISO 22412.

### 2.5. Preparation of Plumbagin-Loaded Nanoemulsions

Plumbagin-loaded nanoemulsions were prepared by low-energy spontaneous emulsification [19]. Briefly, plumbagin was dissolved in Capryol 90 in the range 0.4–4.7% (*w*/*w*) and mixed for 30 min at 25°C. The solution of plumbagin in Capryol 90 was then mixed with a blend of excipients Labrasol/Kolliphor RH 40 (1 : 1 *w*/*w*) at surfactant-cosurfactant to Capryol 90 ratio of 1.35. This organic phase with plumbagin and excipient mixture was mixed on a magnetic stirrer for 10 min at 25°C. Nanoemulsions were then produced by dispersing of the organic phase into deionized water in one step to the final concentration of water, 40.5% (*w*/*w*). Dispersions were vortexed for 10 sec at 25°C.

### 2.6. Physical Stability of Nanoemulsions

Control and plumbagin-loaded nanoemulsion formulations were analyzed for changes in particle size distribution over time. To study stability in simulated physiologic environments, the formulations were dispersed in 0.1 M HCl and 0.01 M sodium phosphate buffer pH 6.8 and pH 7.5, with 100-fold dilution. The particle size distribution was measured at designated time-points by DLS using Zetasizer Nano-ZS (Malvern Instruments) as described above.

### 2.7. Cell Culture

PTEN-P2 murine prostate cancer cell line was previously characterized and kindly supplied by Dr. Wu Laboratory [20]. The cells were grown in phenol red-free RPMI-1640 medium (Sigma) supplemented with 10% (*v*/*v*) heat-inactivated fetal bovine serum, 2 mM L-glutamine, 100 U/ml penicillin 100 *μ*g/ml streptomycin, insulin-selenium-transferrin (5 *μ*g/ml insulin), and 10^−8^ mol/l dihydrotestosterone. Cultures were passaged by dissociation with trypsin (0.05%) and maintained at 37°C in a humidified atmosphere with 5% CO_2_.

### 2.8. In Vitro Cytotoxicity Assay

The cytotoxicity of plumbagin formulations was examined using the MTS tetrazolium compound-based method. PTEN-P2 cells were seeded at a density of 8 × 10^3^ cells/well in 96-well plates in replicates (*n* = 4). Then, 24 h later, the medium was changed for medium containing free plumbagin or plumbagin formulations corresponding to the concentration range of 0-10 *μ*mol/l plumbagin. Free plumbagin control was prepared by dissolving plumbagin in dimethylsulfoxide (DMSO). DMSO was kept at constant concentration (0.1% *v*/*v*) within the tested concentration range of plumbagin. Control formulation without plumbagin was analyzed at the same concentration range. The antiproliferative effect was determined after 24 h incubation using the CellTiter 96 AQueous one solution cell proliferation assay kit according to the manufacturer's instructions (Promega, Madison, WI) by measuring the conversion of (3-(4,5-dimethylthiazol-2-yl)-5-(3-carboxymethoxyphenyl)-2-(4-sulfophenyl)-2*H*-tetrazolium, inner salt) to formazan product. Half-maximal inhibitory concentration (IC_50_) values were interpolated from cytotoxicity curves as the concentration that induced 50% inhibition of the cell growth.

The article "Propylene Glycol Caprylate-Based Nanoemulsion Formulation of Plumbagin: Development and Characterization of Anticancer Activity" was published in 2022. Journal: Biomed Res Int.

## 3. Results

### 3.1. Selection of Excipients and Formulation Development

In order to select the optimal constituents of a nanoemulsion formulation for plumbagin, we first measured the solubility of plumbagin in various lipid-based excipients. As shown in Table 1, excipients based on medium chain glycerides such as Labrasol, Labrafac, and Capmul MCM, or on propylene glycol esters such as Capryol 90, have a remarkably high capacity to solubilize plumbagin. Indeed, plumbagin concentrations in these excipients are higher than 80 mg/ml, reaching 125mg/ml in Labrasol, compared to 50-60 mg/ml range in glyceryl trioleate, Peceol, Span 80, or Span 85. This is much higher than the solubility achieved in organic solvents, which ranges from 22 mg/ml in DMSO to 48 mg/ml in ethyl acetate [10, 11]. It is also higher than the solubility achieved in plant-derived oils, which reaches a maximum of 57.1 mg/ml in sesame oil and is the excipient used in proof-of-efficacy animal studies and first-in-human clinical trial [10, 11].

Based on preformulation studies of the miscibility of various systems of oils and surfactants, their dispersibility in water, and on results of plumbagin solubility shown in Table 1, Capryol 90 (propylene glycol monocaprylate) was selected as an oil phase and Labrasol/Kolliphor RH 40 as a nonionic surfactant/cosurfactant mixture for the development of a new nanoemulsion formulation.

To identify the monophasic, optically isotropic region of the nanoemulsion and to determine the optimal concentration of excipients, a series of mixtures of containing various ratios of Capryol 90 with surfactant Labrasol/cosurfactant Kolliphor RH 40 (1 : 1, *w*/*w*) were prepared. The pseudoternary phase diagram, shown in Figure 2(a), was constructed using progressive water titration as described in Materials and Methods. The established pseudoternary phase diagram was then used to delineate the nanoemulsion domain and the boundary of phases. Samples falling within the nanoemulsion domain appeared translucent whereas mixtures with higher ratios of the Capryol 90 oil phase led to the formation of opalescent coarse dispersions (Figure 2(b)).

The article "Propylene Glycol Caprylate-Based Nanoemulsion Formulation of Plumbagin: Development and Characterization of Anticancer Activity" was published in 2022. Journal: Biomed Res Int.

Aqueous dispersions of samples with different surfactant/cosurfactant-to-oil (S-CoS/O) ratios were further characterized by photon correlation microscopy (PCS) using Zetasizer Nano-ZS (Malvern). PCS, dynamic light scattering based at 173° backscattering angle, was used to estimate the particle size distribution and the polydispersity of each formulation (Figure 3). *Z*-average, an intensity-based harmonic mean determined by method of cumulants, clearly showed dependency on the S-CoS/O (Figure 4). Figures 3 and 4 show that the hydrodynamic diameter fell into the range of nanoemulsions at S − CoS/O > 1.2 with a low polydispersity index (PDI). Analysis of particle size distribution over time for samples with S − CoS/O < 1 showed a very broad size distribution profile and high polydispersity and instability, while formulations in which the S-CoS/O ratio was within the range of 1.35–1.7 showed a narrow PDI and stability of size distribution over time.

### 3.2. Stability of Plumbagin-Loaded Nanoemulsion

The nanoemulsion formulation consisting of an S-CoS/O ratio of 1.35 was selected for further development. Nanoemulsions loaded with increasing amounts of plumbagin (0.4–4.7% *w*/*w*) as well as an “empty” formulation without plumbagin displayed similar particle size distributions immediately after production (Figure 5). Both the control and the plumbagin-loaded nanoemulsions showed retention of size distribution during six months of storage at 25°C (Figure 5(b)), indicating good stability over extended period of time.

Finally, the stability of the nanoemulsions was measured in simulated physiological environments. Results presented in Table 2 showed good retention of particle size for both the control (empty) and the plumbagin-loaded nanoemulsions when dispersed in media that simulate the physiological environment of stomach acid and intestinal fluids.

### 3.3. In Vitro Antiproliferative Activity of Plumbagin-Loaded Nanoemulsion

The cytotoxicity of the plumbagin-loaded nanoemulsion was evaluated by exposing prostate cancer cells PTEN-P2 to increasing dilutions of the formulation with and without plumbagin for 24 h.  Figure 6 demonstrates the dose-dependent cytotoxicity of plumbagin-loaded nanoemulsion compared to the cytotoxicity of free plumbagin. The plumbagin-loaded nanoemulsion formulation displayed higher inhibitory effect on proliferation of PTEN-P2 cells compared to free plumbagin, with IC_50_ 2.5 vs. 4.3 umol·l^−1^, respectively. These findings correlate with an assessment of cell gross morphology, showing that the plumbagin-loaded nanoemulsion formulation induced substantial cell detachment, shrinkage, and cellular damage compared to free plumbagin (Figure 7). Control, drug-free nanoemulsion did not demonstrate notable cytotoxicity in the analyzed range (Figures 6 and 7).

The article "Propylene Glycol Caprylate-Based Nanoemulsion Formulation of Plumbagin: Development and Characterization of Anticancer Activity" was published in 2022. Journal: Biomed Res Int.

## 4. Discussion

The majority of therapeutic chemical entities in drug development have poor aqueous solubility [21, 22], which is a significant challenge limiting potential clinical translation. Recent years have seen a mounting effort to bring new drug solubilization and delivery technologies at an earlier stage of the preclinical development process in order to facilitate successful progression into the clinic [23].

Several drug delivery systems have been explored as carriers to formulate plumbagin and potentially improve its anticancer activity, including niosomes, serum albumin, silica nanoparticles, chitosan, poly (lactic-co-glycolic) acid (PLGA), micelle-based systems, gold nanoparticles, and liposomes [24–30]. While these studies showed promising results, production of most of these formulations is costly and/or requires the use of organic solvents or components that are not biocompatible, which limits their translational application. In order to develop a simple, cost-effective, and scalable formulation, we have focused on a nanoemulsion formulation designed using biocompatible pharmaceutical excipients. Furthermore, nanoemulsion formulations have demonstrated excellent absorption and bioavailability, enhanced penetration of biological membranes, and lower inter- and intraindividual variability in drug pharmacokinetics compared to naked drugs [14, 15]. Last but not least, nanoemulsions are compatible with per oral administration, which is highly desirable as the per oral route results in better patient compliance compared to other routes of administration. In addition, per oral administration does not require hospital stay and therefore is more accessible to patients, especially low-income patients with restricted access to health care, as well as patients living in rural or undeveloped areas.

Our preformulation studies identified medium-chain glyceride-based excipients with a high solubilization capacity for plumbagin. A stable formulation of plumbagin was designed using Capryol 90 as an oil phase and Labrasol/Kolliphor RH40 (1 : 1) as surfactant and cosurfactant. Capryol 90 has been used to develop nanoemulsion-based drug delivery systems with particle size distribution comparable to our formulation [31–33]. The plumbagin-loaded nanoemulsion (30.9 nm *Z*-average, Capryol 90 to Labrasol/Kolliphor 40; 1.35 *w*/*w*) demonstrated good retention of size distribution and narrow polydispersity over extended periods of time, indicating good shelf-life with undemanding temperature requirements that would facilitate manufacturing, storage, and distribution.

The article "Propylene Glycol Caprylate-Based Nanoemulsion Formulation of Plumbagin: Development and Characterization of Anticancer Activity" was published in 2022. Journal: Biomed Res Int.

Retention of nanoparticle size after dispersion in water or media emulating physiological fluids also suggested potential stability in the gastrointestinal tract that would permit optimal absorption in vivo.

It is reasonably expected that plumbagin delivered/released from the nanoemulsion formulation should exhibit its pharmacological activities towards various types of cancer cells as extensively described in literature, since plumbagin has shown no discrimination toward cancer types. Noteworthy, observed cytotoxicity of plumbagin toward PTEN-P2 prostate cancer cells, both as a free drug and in the form of drug-loaded nanoemulsion, was slightly higher compared to standard of care for prostate cancer—docetaxel or other anticancer drugs in development, rapamycin and 17-AAG encapsulated in the poly(ethylene glycol)-block-poly(D,L-lactic acid) (PEG-b-PLA) micelles [34].

In vitro cytotoxicity studies of the plumbagin-loaded nanoemulsion showed a slightly augmented antiproliferative effect of the active pharmaceutical ingredient (plumbagin) against PTEN-P2 prostate cancer cells compared to free drug. This is not attributable to an additive effect of cytotoxicity of individual components, because the control formulation (nanoemulsion without drug) did not exhibit cytotoxicity at equivalent doses. Thus, increased cytotoxicity of the plumbagin nanoemulsion formulation compared to free plumbagin can be attributed to a higher cellular uptake of the nanoparticulate form, to a stabilizing effect of the nanoemulsion on plumbagin, or a combination of both. Indeed, the high particle surface area [15] associated with a high surface to mass ratio due to the small diameter of the nanoparticulate dispersion is expected to increase its interaction with cell surfaces, yielding a higher cellular uptake of plumbagin. Importantly, plumbagin is an *α*, *β*-unsaturated diketone (1,4-naphthoquinone) electrophile capable of undergoing Michael's addition reaction with endogenous nucleophiles [35], including serum albumin [26], and is therefore extremely reactive. Encapsulation of plumbagin in the hydrophobic core of the nanoemulsion would decrease its interaction with nucleophiles before reaching cellular targets. This effect is expected to improve the pharmacokinetic/pharmacodynamic profile of plumbagin when administered in the form of a nanoemulsion.

The article "Propylene Glycol Caprylate-Based Nanoemulsion Formulation of Plumbagin: Development and Characterization of Anticancer Activity" was published in 2022. Journal: Biomed Res Int.

## 5. Conclusion

We have developed a plumbagin-loaded nanoemulsion formulation using lipid-based excipients that are biocompatible and have been used in clinically approved pharmaceutical products. High loading capacity and retention of nanoparticle size over extended time and in a simulated physiological environment as well as *in vitro* anticancer activity indicate that the Capryol 90-based nanoemulsion formulation of plumbagin has significant translational potential.

## Figures and Tables

**Figure 1:** Chemical structure of plumbagin (5-hydroxy-2-methyl-1,4-naphthoquinone or 5-hydroxy-2-methyl-1,4-naphthalenedione, C_11_H_8_O_3_).

**Figure 2:** Pseudoternary phase diagram (a) of Capryol 90, Labrasol/Kolliphor RH 40 (1 : 1), and water at 25°C. The grey area indicates o/w nanoemulsion domain. (b) Shows the samples with different w/w ratio of surfactant–cosurfactant to oil (S–CoS/O) ranging from opalescent coarse emulsions to optically translucent nanoemulsions.

**Figure 3:** Time-dependent intensity-based particle size distribution profiles (hydrodynamic radius, *Z*-average, nm) and polydispersity index (PDI) of Capryol 90-Labrasol/Kolliphor RH 40 (1 : 1) at different surfactant-cosurfactant to oil (S-CoS/O) (*w*/*w*) ratios.

**Figure 4:** Hydrodynamic radius (*Z*-average, nm) and PDI of Capryol 90-Labrasol/Kolliphor RH40(1 : 1) dispersions as a function of surfactant-cosurfactant to oil (S-CoS/O) (*w*/*w*) ratio.

**Figure 5:** Stability of size distribution (hydrodynamic radius over time) of plumbagin-loaded Capryol 90-Labrasol/Kolliphor RH40 (1 : 1) nanoemulsions.

**Figure 6:** *In vitro* antiproliferative activity of plumbagin-loaded nanoemulsion. Effect of free plumbagin (PLBG), plumbagin-loaded nanoemulsion (NE-PL, 4.7% *w*/*w*), and control empty nanoemulsions (NE-C) on cell viability of PTEN-P2 cells was determined in a dose-dependent manner. For control drug-free nanoemulsion, NE-C, the cells were exposed to the same concentration of nanoemulsion without plumbagin. PTEN-P2 cells were incubated with increasing dilutions of formulations for 24 h, and then, % cell viability was determined using cell proliferation assay (MTS).

**Figure 7:** Morphological changes pf PTEN-P2 cells after exposure to plumbagin-loaded nanoemulsions. Bright-field microscopy images show untreated control (a) and cells exposed for 24 h to free plumbagin (4 *μ*mol/l) (b), empty nanoemulsion (c), and plumbagin-loaded (4 *μ*mol/l) nanoemulsion formulation (d).

**Table 1:** Solubility of plumbagin in lipid-based pharmaceutical excipients at 25°C.

Excipient	Plumbagin	
	mg/ml	±SD
Capryol 90 (propylene glycol monocaprylate (type II) NF)	94.6	0.4
Labrasol (caprylocaproyl macrogol-8 glycerides)	125.0	1.2
Labrafil M 1944 CS (oleoyl macrogol-6 glycerides)	82.1	0.5
Labrafac lipophile WL 1349 (caprylic/capric triglyceride IIG)	89.4	0.1
Capmul MCM EP/NF (glycerol monocaprylocaprate, type I)	92.0	0.6
Capmul PG-12 EP/NF (propylene glycol monolaurate)	83.7	0.1
Glyceryl trioleate	58.6	0.3
Peceol (glyceryl monooleate, type 40)	52.0	0.1
Span 80 (Sorbitan monooleate)	53.5	0.5
Span 85 (Sorbitan trioleate)	57.9	0.1

The article "Propylene Glycol Caprylate-Based Nanoemulsion Formulation of Plumbagin: Development and Characterization of Anticancer Activity" was published in 2022. Journal: Biomed Res Int.

**Table 2:** Stability of nanoemulsions in simulated physiological environments. Changes in particle hydrodynamic radius and PDI of control (NE-C, empty) and plumbagin-loaded (NE-PL, 4.7% *w*/*w*) nanoemulsions were monitored by DLS after dispersion in indicated media and incubation for 24 h at 37°C. PDI values are shown in brackets.

Z-average hydrodynamic radius (nm) and PDI in different media				
	Water	HCl 0.1 M	0.01 M NaH_2_PO_4_/Na_2_HPO_4_	
			pH 6.8	pH 7.5
NE-C (control)	32.2 (0.180)	30.6 (0.098)	32.4 (0.173)	33.8 (0.165)
NE-PL (loaded)	30.0 (0.162)	30.1 (0.135)	30.0 (0.142)	31.74 (0.135)

## Data Availability

All data are available at Vaccine Research Institute of San Diego, San Diego Science Center, San Diego, CA.
